The article "Clinical Observation of Ultrasound-Guided Nerve Block Anesthesia on Postoperative Pain Control of Fracture Patients" was published in 2022. Journal: J Healthc Eng.

# Clinical Observation of Ultrasound-Guided Nerve Block Anesthesia on Postoperative Pain Control of Fracture Patients

**DOI:** 10.1155/2022/9510669

**Published:** 2022-04-07

**Authors:** Yong Zhao, Huiwen Zhang, Miaomiao Song

**Affiliations:** ^1^Department of Orthopedic, Shanghai Fengxian District Central Hospital, Shanghai 201400, China; ^2^Department of Anesthesiology, General Hospital of Ningxia Medical University, Yinchuan 750002, China; ^3^Department of Anesthesiology, Shanghai Fengxian District Central Hospital, Shanghai 201400, China

## Abstract

To observe the postoperative pain control and clinical efficacy of ultrasound-guided nerve block anesthesia for patients with tibial fracture. A total of 128 patients with tibial fracture who received surgical treatment in our hospital from October 2020 to April 2021 were selected. The ultrasound guided anesthesia group and general anesthesia group were established by random number table method, with 64 patients in each group. Patients in the ultrasound-guided anesthesia group received ultrasound-guided nerve block anesthesia, and patients in the general anesthesia group received conventional general anesthesia. Observation times anesthetic effect in both groups, changes in hemodynamic parameters, digital pain scale (NRS) score as a result, compared two groups of patients with adverse reactions occur, change of the serum inflammatory factors indicators before and after operation, and USES the Pearson correlation coefficient analysis of the correlation between serum levels of inflammatory factor index and NRS score. The effect of anesthesia, postoperative recovery, directional force recovery, motor block and sensory block time of patients in ultrasound-guided anesthesia group decreased significantly than those in general anesthesia group (all *P* < 0.05). The comparison of MAP, HR and RR at T1 and T2 levels between the two groups was statistically significant (all *P* < 0.05). The changes of MAP, HR and RR in ultrasound guided anesthesia group were more stable than those in general anesthesia group.The NRS scores of patients in both groups showed an increasing trend with the extension of time. The 6 h, 12 h and 24 hNRS scores of patients in the ultrasound guided anesthesia group decreased significantly than those in the general anesthesia group (all *P* < 0.05). The total incidence of adverse reactions in ultrasound guided anesthesia group decreased significantly than that in general anesthesia group (*P* < 0.05).The serum levels of inflammatory factor interleukin-6 (IL-6) and tumor necrosis factor-*α* (TNF-*α*) in 2 groups increased significantly before surgery, and the levels of each index in ultrasound guided anesthesia group decreased significantly than that in general anesthesia group (ALL *P* < 0.05). Pearson correlation coefficient showed that serum IL-6 and TNF-*α* levels were positively correlated with NRS score (all *P* < 0.05). Ultrasound-guided nerve block anesthesia surgery can effectively improve the tibia fracture patients intraoperative anesthetic effect, improve patients with intraoperative and postoperative hemodynamic index of stability, the anesthesia surgery will exert positive effects on patients with postoperative pain control, can reduce the risk in patients with postoperative adverse reactions, reduce the postoperative patients with inflammatory factor activity. In addition, this paper found significant positive correlation between serum inflammatory factors IL-6 and TNF-*α* and NRF score, suggesting that serum IL-6 and TNF-*α* can be monitored for postoperative pain control in patients with tibial fracture, providing reference for improving postoperative treatment plan of patients.

## 1. Introduction

Tibial fracture is a common emergency in orthopedic diseases, and patients are troubled by fracture pain and seriously affect their motor function. Surgical treatment is mostly used in clinical practice, and assisted by efficient anesthesia is particularly important to relieve postoperative pain and promote rapid recovery [1]. The basic principle of preoperative anesthesia method selection is not only to meet the depth of anesthesia required for surgery, but also to ensure anesthesia safety [2]. Previous studies have found that it takes longer for patients to wake up after conventional general anesthesia, and the slow recovery of various postoperative functions may lead to postoperative adverse complications, and the range of hemodynamic changes in patients is relatively obvious. Peripheral regional nerve block has attracted more attention because of its small interference to respiration and circulation, relatively few contraindications and complications [3]. The key to nerve block analgesia is to ensure sufficient diffusion of local anesthetic drugs in the nerve region, among which ultrasound guidance is one of the commonly used methods of block localization [4]. Ultrasound-guided nerve block technology uses ultrasound to change the nerve block technology of blind exploration into the nerve block technology of visual, dynamic and continuous observation, and improve the safety of nerve block anesthesia.

In order to further explore the clinical efficacy and pain control mechanism of ultrasonic-guided nerve block anesthesia for patients with fracture, patients with tibial fracture in our hospital were selected as the research objects and group observation was carried out to explore the anesthesia effect and pain control in tibial fracture surgery, to observe its clinical effect and research value.

## 2. Data and Methods

### 2.1. General Data

A total of 128 patients with tibial fracture who received surgical treatment in our hospital from October 2020 to April 2021 were selected. Ultrasound guided anesthesia group and general anesthesia group were established according to random number table method, with 64 patients in each group. There were 36 males and 28 females in the ultrasound guided anesthesia group, aged from 27 to 58 years, with an average of (43.18 ± 5.52) years. 33 patients were grade I and 31 were grade II, according to the Classification of American Society of Anesthesiologists (ASA). In the nerve block anesthesia group, there were 34 males and 30 females, aged from 29 to 60 years old, with an average of (44.02 ± 5.60) years old. ASA grading showed 35 cases of grade I and 29 cases of grade II. There were no significant statistical differences in gender, age, ASA grade and other general data between groups (all *P* > 0.05), which confirmed that the comparison between groups was scientific and reasonable. Inclusion criteria: (1) patients with tibial fracture diagnosed by imaging detection and clinical diagnosis [5]; (2) complete clinicopathological data; (3) no anesthesia related contraindications; (4) Patients have high cooperation, clear consciousness, and no cognitive impairment, and understand and give informed consent to this paper. Exclusion criteria: (1) patients with blood system diseases or signs of coagulopathy; (2) Patients with a history of chronic pain or signs of peripheral neuropathy; (3) persons with serious organic dysfunction such as liver and kidney; (4) Skin infection or inflammatory lesions at the injection site; (5) Poor compliance or incomplete cost of researchers for various reasons.

### 2.2. Methods

#### 2.2.1. Anesthesia Methods

Patients in general anesthesia group were induced by general anesthesia, and all patients in the group received 0.08 mg/kg midazolam before surgery (Jiangsu Nhwa Pharmaceutical Co., Ltd, Batch Number: Then 0.03 mg/kg midazolam, 3 *μ*g/kg fentanyl (manufacturer: Yichang Renfu Pharmaceutical Co., LTD., Batch No.: H42022076), 1.5 mg/kg propofol (Xi ‘an Libon Pharmaceutical Co., LTD., Batch No.: National Medicine Approval H19990282), 0.6 mg/kg rocuronium (Zhejiang Xianju Pharmaceutical Co., Ltd., Batch Number: National medicine approval H20093186) was injected intravenously. During induction of general anesthesia, patients' vital signs were monitored to observe whether there was stimulation response or unconsciousness. After confirmation of no adverse conditions, the disposable double-tube laryngeal mask was placed and connected with the ventilator. In the ultrasound guided anesthesia group, ultrasound guided nerve block anesthesia was performed after induction of general anesthesia. Patients were placed in supine position and their groin was routinely disinfected. GELOGIQ E9 color Doppler ultrasound diagnosis system was used to place a portable ultrasound probe at the pulse point of the groin femoral artery, and 15 mL 0.375% ropivacaine (manufacturer: Chenxin Pharmaceutical Co., LTD., Batch Number: The femoral nerve block was completed by injection around the femoral nerve, then the affected limb was raised, the popliteal fossa skin was routinely disinfected, the ultrasonic probe was placed near the popliteal transverse veins, the probe was fixed at the distal branch of the sciatic nerve, and 15 mL 0.375% ropivaine was injected by in-plane technique. On this basis, sciatic nerve block was completed, and it could be observed from the ultrasound image that the nerve tracts of the patient were infiltrated by drug solution. For the nerve tracts that were not infiltrated successfully, the position of the needle tip was changed to get close to the nerve, and then the drug was injected until the nerve tracts were completely infiltrated by drug solution.

#### 2.2.2. Detection Method of Serum Inflammatory Factors

8 mL fasting venous blood was collected from all patients in the morning before and after surgery, centrifuge parameters were set to 3500 r/min, centrifugation radius was 10 cm, centrifugation for 10 min, then the supernatant was taken, and the serum inflammatory factors were measured by ELISA. Kit was purchased from Shanghai Kehua Bio-Engineering Co., Ltd.

### 2.3. Observation Indicators

(1) Anesthesia effect at each time period was compared between the two groups; (2) Changes of intraoperative and postoperative hemodynamic indexes, including preoperative anesthesia (T0), Mean Arterial Pressure (MAP) and Heart Rate (T3) 10 min after puncture (T1), skin dissection time (T2). HR) and Respiratory Rate (RR); (3) The Numerical Rating Scale (NRS) scores of patients in the two groups at various postoperative periods were compared, including 6 h, 12 h and 24 h after surgery; (4) Adverse reactions, including chills, nausea and vomiting, and urinary retention, were compared between the two groups; (5) Changes of serum inflammatory factors, including IL-6 and TNF-*α* levels, were compared between the two groups before and after surgery. (6) Pearson correlation coefficient was used to analyze the correlation between serum inflammatory factors IL-6 and TNF-*α* and NRS score.

Postoperative pain was assessed by NRS scale [6]. Patients described pain intensity on a scale of 0 to 10, with a higher pain score indicating more severe pain. 0 is no pain, 1 to 3 is mild pain that does not affect sleep quality, 4 to 6 is moderate pain, 7 to 9 is severe pain that has seriously affected sleep quality, and 10 is severe pain.

### 2.4. Statistical Methods

SPSS 26.0 software was used for statistical analysis of the paper data, and the measurement data were verified. After confirming that the data were normally distributed, mean ± standard deviation($\bar{x}$ ± *s*)was used to represent the data. Two independent sample *T*-test and paired *T*-test were performed. (*n*, %) was used to represent the counting data involved, *x*^2^ test was used for data differences between groups and effective analysis was completed, repeated measure anOVA was used for multi-group comparison, spherical test (Mauchly) was used for data comparison at different time points within the group, *P* > 0.05 indicated that the covariance matrix was full of football symmetry. Pearson correlation coefficient was used to analyze the correlation between the changes of serum inflammatory factors IL-6 and TNF-*α* and NRS score, *P* < 0.05 confirmed that the difference was statistically significant.

## 3. Experimental Results

### 3.1. Comparison of Anesthesia Effects in Each Time Period between the Two Groups

The time of anesthesia onset, postoperative recovery, directional force recovery, motor block and sensory block in the ultrasound-guided anesthesia group decreased significantly than that in the general anesthesia group (all *P* < 0.05), as shown in Table 1.

### 3.2. Comparison of Hemodynamic Indexes at Different Time Periods between the Two Groups

There were no significant differences in MAP, HR and RR indexes between the two groups at T0 and T3 (all *P* > 0.05), but there were significant differences at T1 and T2 (all *P* < 0.05). In addition, MAP, HR and RR changes in each time period in the ultrasound guided anesthesia group were smaller than those in the general anesthesia group, as shown in Table 2.

### 3.3. Comparison of NRS Scores between the Two Groups at Each Time Point after Surgery

NRS scores in both groups showed a significant upward trend as time went on, but 6 h, 12 h and 24 hNRS scores in the ultrasound-guided anesthesia group were significantly lower than those in the general anesthesia group (all *P* < 0.05), as shown in Table 3.

### 3.4. Comparison of Adverse Reactions between the Two Groups

The incidence of chills, nausea/vomiting and urinary retention in the ultrasound guided anesthesia group was lower than that in the general anesthesia group, and the total incidence was significantly lower than that in the general anesthesia group (*P* < 0.05), as shown in Table 4.

### 3.5. Comparison of Changes in Serum Inflammatory Factor Levels before and after Surgery between the Two Groups

There were no significant differences in serum IL-6 and TNF-*α* levels between the two groups before surgery (all *P* > 0.05). Indexes in both groups increased significantly after surgery than before, and indexes in the ultrasound-guided anesthesia group were significantly lower than those in the general anesthesia group (all *P* < 0.05), as shown in Table 5.

### 3.6. Analysis of the Correlation between Changes of Serum Inflammatory Factors and NRS Score

Pearson correlation coefficient showed that serum inflammatory factors IL-6 and TNF-*α* were significantly positively correlated with NRS score (all *P* < 0.05).  Figure 1 is correlation between serum IL-6 and NRS score.  Figure 2 displays correlation between serum TNF-*α* and NRS score.

## 4. Experimental Result Discussion

The occurrence of tibial fracture requires surgical treatment as soon as possible. Although conventional general anesthesia has a definite curative effect, it may cause large fluctuations in hemodynamics of patients during anesthesia, increasing the risk of the whole operation and adversely affecting the prognosis of patients to some extent [7]. In recent years, the technical level in the medical field has made continuous progress, promoting the development of medical equipment in the direction of precision and visualization. Ultrasound guidance technology has been widely used in clinical surgery and achieved satisfactory results [8]. Ultrasound guided precision positioning of target nerve, accurately into nerve conduits, under the condition of the optimal anesthetic effect, is helpful to avoid damage when the needles are vascular nerves, can make the anesthetic solution package around the target nerves, to improve the accuracy of the block and the success rate, the maximum extent to reduce the risk of peripheral nerve and vascular injury, It has been widely used in lower limb nerve block surgery at present. Ultrasound-guided nerve block combined with general anesthesia is monitored by ultrasound instrument, and general anesthesia is performed after the sciatic nerve in the popliteal fossa of the patient's affected limb is blocked with proportional local anesthesia [9]. The use of ultrasound equipment helps the anesthesiologist to quickly complete precise positioning during nerve block anesthesia, thus reducing the degree of nerve damage in patients and having a positive effect on alleviating postoperative pain [10].

This paper result shows that ultrasonic guided nerve block anesthesia to shorten the anesthesia effect, recovery of awakening, directional force, motor block and block time has obvious utility, and have less effect on the level of patients with hemodynamic indicators, prompt the anesthesia operation of promoting blood flow dynamics in patients with stable with a high utility, effectively improve the safety of fracture surgery. It is helpful for the smooth operation of patients and has positive significance for the rapid postoperative recovery of patients, which is similar to the research results of Yang Peng et al. [11]. Analysis of the reason may be the accuracy of ultrasound guided nerve block positioning make accurate injection target plexus anesthesia drugs and obvious effect, reduce the intraoperative should at the same time also can effectively control the local anesthesia drug dosage, effectively restrain the patient's stress response and reduce the risk of patients after anesthesia complications, the efficacy and safety of clinical has higher [12].

This paper observed and analyzed the pain degree and changes in serum inflammatory factors IL-6 and TNF-*α* levels of patients in the two groups at each time after surgery. The comparison showed that postoperative NRS score and serum factor levels of patients in the neuro-guided anesthesia group were significantly lower than those in the general anesthesia group, which was similar to the results of Liu et al. [13]. Regular general anesthesia has certain blindness, explore sex during anesthesia for patients with peripheral nerve and vascular damage degree is more obvious, under the guidance of ultrasound can clearly show the target neural structures, needle and local anesthetics diffusion situation, improve the effect of blocking, reducing the body injury, may be due to the ultrasonic guided nerve block anesthesia, Patients' body's response to surgical trauma is reduced, which helps to inhibit the activation of inflammatory factors and alleviate trauma [14, 15]. In order to further explore the pain control mechanism of tibial fracture patients, this paper used Pearson correlation coefficient to analyze serum inflammatory factors and NRS score, and showed that serum IL-6 and TNF-*α* were significantly positively correlated with NRS score, suggesting that increased serum TNF-*α* and IL-6 levels may be closely related to anesthesia effect. Therefore, it is suggested that serum TNF-*α* and IL-6 levels can be monitored during the evaluation of postoperative pain in patients with fracture, providing a new direction for the subsequent pain management and control of patients and the formulation of postoperative rapid rehabilitation programs.

The results and corresponding conclusions of this paper are shown above, which have certain reference value for providing better clinical anesthesia program for patients with tibial fracture, but there are still some deficiencies. First sample size selection is less and short survey time setting may affect the scientific nature of this paper follow-up paper should expand the scope of sample size and sample, and for patients with postoperative pain control and quick recovery mechanism to further explore, enlarge the research of relevant indicators, to further improve the results of the paper of science degrees and accuracy.

## 5. Conclusion

In conclusion, ultrasound-guided nerve block anesthesia has a positive effect on the improvement of clinical safety in fracture surgery, the hemodynamics of patients is more stable, the time to wake up and the time to independent recovery is effectively shortened, and the incidence of adverse reactions is reduced, which confirms its good blocking effect and high clinical application value. In addition, this paper found significant correlation between serum inflammatory factors IL-6 and TNF-*α* and patients' pain degree, which is of great significance for follow-up clinical monitoring of fracture patients after surgery, achieving accurate pain assessment and improving pain management programs.

## 6. Clinical Registration Number

KY-2022-2016-01.

## Figures and Tables

**Figure 1:** Correlation between serum IL-6 and NRS score.

**Figure 2:** Correlation between serum TNF-*α* and NRS score.

**Table 1:** Comparison of anesthesia effect between the two groups at different time periods (min, $\bar{x}$ ± *s*).

Group	Time of onset of anesthesia	Postoperative recovery time	Recovery time of directional force	Onset time of motor block	Onset time of sensory block
Ultrasound guided anesthesia group (*n* = 64)	6.96 ± 2.88	13.75 ± 2.87	22.13 ± 3.24	15.92 ± 2.02	14.95 ± 1.79
General anesthesia group (*n* = 64)	8.84 ± 3.15	17.92 ± 3.11	26.47 ± 3.66	21.76 ± 2.64	20.01 ± 1.93
*t*	3.524	7.883	7.103	14.055	15.378
*P*	<0.001	<0.001	<0.001	<0.001	<0.001

**Table 2:** Comparison of changes in hemodynamic indexes between the two groups at different time periods ($\bar{x}$ ± *s*).

Indicators	Group	T0	T1	T2	T3
MAP (mmHg)	Ultrasound guided anesthesia group (*n* = 64)	95.18 ± 4.13	92.56 ± 3.92^*∗*^	93.92 ± 4.25	95.14 ± 3.71^#△^
	General anesthesia group (*n* = 64)	95.03 ± 3.86	86.51 ± 4.33^*∗*^	88.39 ± 4.97^*∗*^^#^	95.11 ± 4.06^#△^
	*t*	0.212	8.286	6.765	0.335
	*P*	0.832	<0.001	<0.001	0.739
	Between groups	*F* = 3.541, *P*=0.001			
	Different points in time	*F* = 2.224, *P*=0.001			
	Between groups • different time points	*F* = 3.343, *P*=0.001			
HR (times/min)	Ultrasound guided anesthesia group (*n* = 64)	81.13 ± 4.32	79.56 ± 4.29^*∗*^	80.42 ± 4.31	80.95 ± 4.16
	General anesthesia group (*n* = 64)	81.87 ± 4.28	75.64 ± 4.17^*∗*^	76.37 ± 4.52^*∗*^^#^	81.24 ± 4.19^#△^
	*t*	0.973	5.242	5.188	0.393
	*P*	0.332	<0.001	<0.001	0.695
	Between groups	*F* = 3.421, *P*=0.001			
	Different points in time	*F* = 2.564, *P*=0.001			
	Between groups · different time points	*F* = 3.112, *P*=0.001			
RR (times/min)	Ultrasound guided anesthesia group (*n* = 64)	16.19 ± 1.17	15.53 ± 1.05^*∗*^	15.82 ± 1.21	15.88 ± 1.12
	General anesthesia group (*n* = 64)	16.04 ± 1.08	12.79 ± 1.07^*∗*^	13.51 ± 1.13^*∗*^^#^	15.92 ± 1.04^#△^
	*t*	0.754	14.622	11.162	0.209
	*P*	0.452	<0.001	<0.001	0.834
	Between groups	*F* = 3.175, *P*=0.001			
	Different points in time	*F* = 2.327, *P*=0.001			
	Between groups · different time points	*F* = 2.865, *P*=0.001			

Note. ^*∗*^represents *P* < 0.05 compared with T0; #represents *P* < 0.05 compared with T1; △represents *P* < 0.05 compared with T2.

**Table 3:** Comparison of NRS scores between the two groups at each postoperative time ($\bar{x}$ ± *s*).

Group	Before the operation	6 h after surgery	12 h after surgery	24 h after surgery
Ultrasound guided anesthesia group (*n* = 64)	0.63 ± 0.06	0.82 ± 0.11^*∗*^	1.28 ± 0.42^*∗*^^#^	2.43 ± 0.67^*∗*^^#△^
General anesthesia group (*n* = 64)	0.65 ± 0.07	1.08 ± 0.23^*∗*^	2.17 ± 0.58^*∗*^^#^	3.52 ± 0.71^*∗*^^#△^
*t*	1.735	13.179	9.943	8.932
*P*	0.085	<0.001	<0.001	<0.001
Between groups	*F* = 5.513, *P*=0.001			
Different points in time	*F* = 5.287, *P*=0.001			
Between groups · different time points	*F* = 4.628, *P*=0.001			

Note: ^*∗*^represents *P* < 0.05 compared with preoperative; # represents *P* < 0.05 compared with 6 h after surgery; △ represents *P* < 0.05 compared with 12 h after surgery.

**Table 4:** Comparison of incidence of adverse reactions between the two groups (*n*, %).

Group	Chills	Nausea/vomiting	Urinary retention	Total incidence of adverse reactions
Ultrasound guided anesthesia group (*n* = 64)	3 (4.69)	1 (1.56)	0 (0.00)	4 (6.25)
General anesthesia group (*n* = 64)	5 (7.81)	7 (10.94)	3 (4.69)	15 (23.43)
*x* ^2^	—	—	—	7.479
*P*	—	—	—	0.006

**Table 5:** Comparison of changes in serum inflammatory factors in the two groups before and after surgery.

Group	IL-6		TNF-*α*	
	Before the operation	After the operation	Before the operation	After the operation
Ultrasound guided anesthesia group (*n* = 64)	4.36 ± 1.87	7.33 ± 1.92^*∗*^	5.18 ± 1.64	7.98 ± 2.03
General anesthesia group (*n* = 64)	4.25 ± 1.75	11.34 ± 2.41^*∗*^	5.25 ± 1.69	14.67 ± 2.54
*t*	0.375	10.411	0.238	16.460
*P*	0.708	<0.001	0.812	<0.001

Note: ^*∗*^represents comparison with preoperative, *P* < 0.05.

## Data Availability

The data used to support the findings of this paper are available from the author upon request.
